The article "Footballer Action Tracking and Intervention Using Deep Learning Algorithm" was retracted in 2023. Reasons: signs of a paper mill; suspected computer-generated content; unreliable results or conclusions; lack of ethics approval or compliance.

# Footballer Action Tracking and Intervention Using Deep Learning Algorithm

**DOI:** 10.1155/2021/5518806

**Published:** 2021-03-15

**Authors:** Guanghui Yang, Lijun Wang, Xiaofeng Xu, Jixiang Xia

**Affiliations:** ^1^School of Physical Education, Yanshan University, Qinhuangdao, Hebei 066004, China; ^2^Institute of Physical Education and Health, Yulin Normal University, Yulin 537000, China; ^3^Department of Physical Education, North China University of Science and Technology, Tangshan, Hebei 063000, China; ^4^School of Basic Sciences for Aviation, Naval Aviation University, Yantai, Shandong 264001, China

## Abstract

Fédération Internationale de Football Association is the governing body of the football world cup. The international tournament of football requires extensive training of all football players and athletes. In the training process of footballers, players and coaches recognize the training actions completed by footballers. The training actions are compared with standard actions, calculate losses, and scientifically intervene in the training processes. This intervention is important for better results during the training sessions. Coaches must determine and confirm that every action performed by the footballers meets the minimum standards. It is because the actions of individual players are performed quickly; as a result, the coach's eye may not produce accurate results as human activities are prone to errors. Therefore, this paper designs and develops a footballer's motion and gesture recognition and intervention algorithm using a convolutional neural network (CNN). In this proposed algorithm, initially, texture features and HSV features of the footballer's posture image are extracted and then a dual-channel CNN is constructed. Each characteristic is extracted separately, and the output of the dual-channel network is combined. Finally, the obtained results are passed from a fully connected CNN to estimate and construct the posture image of the footballer. This article performs experimental testing and comparative analysis on a wide range of data and also conducts ablation studies. The experimental work shows that the proposed algorithm achieves better performance results.

## 1. Introduction

Athletes and footballers' action gesture estimation is a widely used branch of computer vision and machine learning [1]. It has a variety of applications which include pose recognition that is dependent on human body modeling. The use of the three-dimensional (3D) human pose recognition and activity recognition technology has been adopted in the literature [2, 3]. Footballer action recognition is an important type of human pose estimation and recognition. Human pose recognition is the identification and location of important points of human targets in the image. The deep convolutional neural network (CNN) has the capability to solve the problem of human pose recognition. The methods of human pose recognition are mainly divided into two parts: top-down method and bottom-up method. The top-down method refers to first detecting the human target, then using the target bounding box [4] to locate, and finally using the single-person estimation method to locate all the joints of the human body. On the other hand, the bottom-up method refers to locating all the joints and positions of the joints, then distinguishing the subordinate targets of the joints, and finally assembling the joints into a complete human body posture [5]. The former is suitable for sparse personnel targets, and the latter is suitable for dense personnel targets.

In literature, the sport training of athlete's action recognition and intervention mechanisms are studied [6–10]. In [6], a depth map method is proposed that is based on local feature recognition. This method uses an extensible graphic model to explicitly implement modeling actions and is based on comparison with the action recognition method of dimensional contour, which produces a better recognition effect. In [10], the authors recommended a global descriptor that considers the direction and size of each body part. In this descriptor, a 3D grid is placed around the person, and the grid is used for motion recognition. In [11], Hadfield et al. recommended a new local motion descriptor of the RGBD video sequence. In this work, a description symbol encodes the extraction of three-dimensional directions from evenly spaced regions to realize action recognition.

In the football player training environment, the coach recognizes the difficult movements completed by the athletes and compares them with standard actions, calculates the loss, and scientifically intervenes in the training process. The coach must identify and confirm that every movement performed by the athlete meets the minimum standards [12–15]. Since athlete's movements are basically completed instantly, the coach recognition experience is prone to errors due to loss of attention and attraction. An example of footballer pose estimation and tracking is shown in Figure 1. As a result, a high-speed camera is needed to take pictures of athlete's movements during training. Therefore, this paper designs and develops an athlete's action recognition and intervention using deep learning [16–21] and big data analytics. In the proposed mechanism massive motion image data is collected, deep CNN is applied for motion recognition that assists the coach to calculate the loss of motion deviation, make corrections, and intervene based on the accurate recognition results. The main contributions of this paper are as follows:

1. The proposed algorithm extracted hue saturation value (HSV) and texture features from action images of athletes and constructed a novel dual-channel CNN. The dual-channel convolutional extraction and fusion features effectively improved the accuracy of action recognition.
2. In the proposed algorithm, a deep learning method is applied that uses big data to recognize the athlete's gesture recognition, which achieves gratifying results.
3. Finally, the proposed scheme has been extensively tested on comparative experiments and ablation studies, which can provide a scientific basis for football coaches to formulate a reasonable training plan.

The rest of the paper is organized as follows: In Section 2, a literature review is studied in detail, while Section 3 provides the detailed methodology.  Section 4 provides detailed results and discussion. Finally, the paper is concluded in Section 5.

## 2. Literature Review

Alexander et al. [22] recommended a method of combining convolutional neural networks and cascades. Through basic estimation, the coordinate of a node is obtained, then the corresponding partial image is obtained through the coordinate, and the partial image is used to achieve higher accuracy. The original image with a lower rate has a poorer effect. At the same time, due to the cascade method, the coordinates of each node need to be subjected to repeated convolution operations. To solve the above limitations, Varun et al. [23] recommended a framework based on Convolutional Pose Machines (CPM), which is applied to human body pose estimation using a neural network to extract spatial information, texture information, and spatial constraint relationship. In the same network, multiscale processing of input feature maps and response maps can not only ensure accuracy but also consider the distance relationship between various parts.

The human pose recognition based on a static frame relies on spatial information and it is very hard to address the problem of human body occlusion and continuous human motion estimation [24]. As a result, Ding et al. [25] recommended a new method on the basis of the relative posture problem of the dual-view minimum case with the homography of the known gravity direction. This is because mobile phones and smart devices have accelerometers and can measure the gravity vector. It also explored the rank 1 constraint of the difference between the Euclidean matrix and the corresponding rotation, proposed an effective two-step method to solve the calibration and semicalibration problems, and obtained satisfactory results. In [26], Kim et al. proposed a method to estimate an individual's posture by analyzing the projection of depth and ridge data using a convolutional neural network, which represents the local maximum in the distance transformation map. With the purpose of making full use of the 3D information of depth points, a method of projecting depth and ridge data in various directions is also proposed. The proposed projection method can decrease the loss of 3D information, the ridge data can avoid joint drift, and CNN can improve the positioning accuracy [22].

In view of the above research, the literature proves that the convolutional neural network has an excellent performance in human body posture, which is better than traditional image processing algorithms. This is the reason why the sued of dual-channel convolutional neural network has numerous advantages.

## 3. Methodology

The architectural flow chart of our proposed algorithm is shown in Figure 2. In this architecture, initially, we extract texture and HSV features from the athlete's action images. Then, a two-channel convolutional neural network is constructed from the obtained features, which is divided into two groups. One group is input with texture features, the other group is input with HSV features, and the outputs of the two groups of convolutional neural networks are combined to obtain global features. Finally, through the fully connected layer, the athlete's posture is estimated.

### 3.1. Feature Extraction

We first extracted texture features (TF) and HSV features as both sets of features will help to improve the performance of the pose estimation. Following is a detailed description of features' extraction and utilization.

#### 3.1.1. Texture Features

Texture is the natural feature of the surface of the target object in the image. It describes the spatial distribution of gray levels between image pixels and image fields and does not change the visibility of the image due to the intensity of light. Therefore, we extracted the texture features of the football athlete's training posture images by calculating the following equation:

(1) $$\begin{array}{c} \text{TF}\left(m_{c},n_{c}\right)=\sum_{P=0}^{P-1}2^{P}s\left(i_{p}-i_{c}\right),s\left(m\right)=\left\{\begin{array}{cc} 1 & m\geq 0\\ 0 & m<0 \end{array}\right\}, \end{array}$$

where (*m*_*c*_, *n*_*c*_) is the central pixel, *i*_*c*_ is the brightness of the point, *i*_*p*_ is the brightness of the adjacent pixels, and *s* is the sign function.

In a 3 × 3 window, we take the central pixel of the window as the threshold and compare the gray value of the adjacent 8 pixels with it. When the surrounding pixel value is greater than the central pixel value, the position of the pixel is marked as 1; otherwise, it is 0. The vector block composed of 1 and 0 is the set of extracted texture features.

#### 3.1.2. HSV Features

The color characteristics of the image hardly depend on the size, direction, and viewing angle of the image itself. Therefore, we choose the HSV feature as one of the features of the footballer's action image. Let (*R*, *G*, *B*) be the red, green, and blue coordinates of a color, respectively; we first normalize it to a real number between 0 and 1. This can be calculated using the following equation:

(2) $$\begin{array}{c} \left\{\begin{array}{c} r=\frac{R}{255},\\ g=\frac{G}{255},\\ b=\frac{B}{255}. \end{array}\right. \end{array}$$

Let max value be equivalent to the largest values of *R*, *G*, and *B* and min be equal to the smallest of these values. Through the following equations, we calculated the hue (*H*), saturation (*S*), and value (*V*):

(3) $$\begin{array}{c} H=\left\{\begin{array}{cc} 0^{{}^{\circ}} & \Delta =0\\ 60^{{}^{\circ}}\times \frac{G-B}{\Delta }+0^{{}^{\circ}} & \max=R\text{ and }G\geq B,\\ 60^{{}^{\circ}}\times \frac{G-B}{\Delta }+360^{{}^{\circ}} & \max=R\text{ and }G<B,\\ 60^{{}^{\circ}}\times \frac{B-R}{\Delta }+120^{{}^{\circ}} & \max=G,\\ 60^{{}^{\circ}}\times \frac{R-G}{\Delta }+240^{{}^{\circ}} & \max=B, \end{array}\right.\\ S=\left\{\begin{array}{cc} 0 & \text{if }\max=0,\\ \left(\Delta /\max\right)=1-\left(\min/\max\right) & \text{otherwise} \end{array}\right.\\ V=\max. \end{array}$$

The above equation outputs RGB features as HSV features. The output new vector block will be input into our proposed algorithm as a feature sequence.

### 3.2. Dual-Channel CNN

The network structure of the dual-channel model, which is similar to the usual neural network and includes a lot of convolutional layers, ReLU layers, and pooling layers is shown in Figure 2. The two channels in the input data, respectively, store the TF feature and the HSV feature. The data of the two channels are input to the network for processing together. The model does not distinguish between global and local for each image block. The network uses the two sets of feature information provided by the two image blocks from the beginning to distinguish the estimated coordinates. The final 2-dimensional output of the fully connected layer of the proposed algorithm is the pose point.

#### 3.2.1. Convolutional Neural Network

A convolutional neural network (ConvNet/CNN) is a deep learning algorithm [27–31] that uses an input image, assigning different weights to various aspects of the image for differentiating purpose. It uses multiple steps; for example, the preprocessing step uses low CNN in regard to other classification algorithms as shown in Figure 3. In the other steps, the ConvNets are trained so that they learn the characteristics of the upcoming inputs. The diagrammatic representation of the CNN is similar to the connectivity-pattern of neurons in the human brain. In other words, CNN is a feedforward neural network with deep structure and convolutional calculation built by imitating the mechanism of human visual perception. CNN has the ability to extract features and can classify the input information according to the hierarchical structure of the input information for translation invariance. The convolution kernel parameter sharing in the hidden layer and the sparsity of the connections between the layers enable CNN to learn spatial features such as pixels and audio with a small amount of calculation, and the effect is stable and there is no additional requirement for data preprocessing.

The different layers of the CNN are shown in Figure 3: the input layer, convolutional layer, pooling layer, and output layer. These layers are described in detail below.

*Input Layer*. The input layer of CNN can handle data of multiple dimensions. One-dimensional convolutional neural networks can process one-dimensional or two-dimensional input data, usually time series or spectrum sampling, whereas 2D convolutional neural networks receive 3D input, usually color images, and the 3D neural networks receive 4D input data, generally color image or video data containing transparent channels. The input layer often preprocesses the original image, including deaveraging, normalization, and whitening (principle component analysis). The purpose of deaveraging is to center all the dimensions of the input data with zero values, while the aim of normalization is to decrease the difficulties caused by the difference in the value range of the data of each dimension. The job of PCA and whitening is to reduce the input data, the dimensions, and the amplitude of each feature axis of the normalized data, respectively.

*Convolutional Layer*. The convolutional layer is the core layer of the CNN, as evident from its name. In the convolutional layer, there are two important operations, local association and sliding window. According to Figure 4, local association means that each neuron represents a filter where each filter calculates the local data, and the sliding window is used to monitor the sliding of the window. The red box in Figure 4 represents a sliding window of the same size and the length of each backward movement of the sliding window, which is called the stride. The convolutional layer extracts local features of the sliding window size through the filter each time. If the step size is too large or the sliding window is too large, most of the part is filled with 0.

*Pooling Layer*. The pooling layer is used to compare the amount of data and the number of parameters to reduce the impact of overfitting. The two commonly used pooling layers include the maximum pooling layer and average pooling layer. These layers determine the most activated presence and the average presence of a feature, respectively. The pooling layer is a newly added layer after the convolutional layer, particularly, when ReLU is applied to the feature sets.

*Output Layer*. The output layer is a fully connected layer, which is used to label the output data. In a fully connected neural with various hidden layers, the output layer gets the output of hidden layers as inputs, performs processing on it using its neurons, and generates the final output.

## 4. Experiments and Results

In this article, we collected 2000 training images of football athlete action images from the Leeds Sports Pose dataset and annotated 14 joints. Those images are challenging due to the different appearances and strong sharpness. The images in the Leeds Sports Pose dataset have been scaled so that the most prominent figures are approximately 150 pixels tall. Although each image in Leeds Sports Pose may contain multiple people, standard preprocessing for human detection has been performed to extract a single person. We use the subimages of these detected individuals as training and testing samples. In this way, the training and testing data contains only one person; in the testing phase, we only use the entire image (for the Leeds Sports Pose dataset, this means the entire subimage of a person) as a body patch.

### 4.1. Evaluation Methods

The pose estimation can be measured by using various metrics, such as the percentage of detected joints and object key point similarity (OKS). In this paper, we have used the OKS metric calculated using equation (6), which is the evaluation index of the commonly used human bone key point detection algorithm. This index is inspired by the intersection over union (IoU) index in target detection. The purpose is to calculate the truth value and predict the similarity of the key points of the human body using the following equation:

(4) $$\begin{array}{c} {\text{OKS}}_{p}=\frac{\sum_{i}\exp\left\{-d_{pi}^{2}/2S_{p}^{2}\sigma_{i}^{2}\delta \left(v_{pi}>0\right)\right\}}{\sum_{i}\delta \left(v_{pi}>0\right)}, \end{array}$$

where *p* represents the person with id *p* among all ground truth pedestrians in the current picture, *p* € (0, M), and *M* represents the number of pedestrians in the current picture. Since the training and test data contain only one person, *M* here is set to 1, and *i* represents the key point with DI *i*. *d*_*pi*_ represents the Euclidean distance between the key point with ID *i* in the set of key points currently detected and the key point with ID *p* in the ground truth pedestrian:

(5) $$\begin{array}{c} d_{pi}=\sqrt{\left(x_{i}^{∼}-x_{pi}\right)\left(y_{i}^{∼}-y_{pi}\right)}, \end{array}$$

where (*x*_*i*_^∼^, *y*_*i*_^∼^) is the current key point detection result, (*x*_*i*_, *y*_*i*_) is the ground truth. *S*_*p*_ represents the scale factor of the person with id *p* in the ground truth pedestrian, and its value is the square root of the area of the pedestrian detection frame:

(6) $$\begin{array}{c} S_{p}=\sqrt{wh}, \end{array}$$

where *w* and *h* are the width and height of the detection frame and *σ*_*i*_ represents the key point normalization factor of type *i*. This factor is the standard deviation between the ground truth key points in all the sample sets and the true value manually marked, *v*_*pi*_ represents the visibility of the *i* key points of the pedestrian with ID *p* in the ground truth, *δ*(*∗*) means if the condition ^*∗*^ holds, then *δ*(*∗*)=1; otherwise, *δ*(*∗*)=0.

Average precision (AP) is used to calculate the accuracy percentage of the test set. Single-person pose estimation: only one pedestrian is estimated at a time, that is, *M*=1 in the oks indicator, so the ground truth in a picture is a pedestrian (GT), and a set of key points will be obtained after the key point detection of this pedestrian (DT); finally calculate the similarity oks between GT and DT as a scalar, then artificially give a threshold T, and finally AP can be calculated from the oks of all pictures:

(7) $$\begin{array}{c} \text{AP}=\frac{\sum_{p}\delta \left(oks_{p}>T\right)}{\sum_{p}1}. \end{array}$$

Percentage of correct parts (PCP): if the key distance between the positions of the two joint points and the real limb reaches at most half the length of the real limb, the joint point is considered to be correctly predicted.

### 4.2. Experimental Results of Different Methods

To fully verify the algorithm in this paper and make an objective comparison, all experiments are carried out in the same environment and the same parameters are used. Using this parameter, the proposed model is compared with the Dantone and Kim [32], Tian et al. [33], Johnson et al. [34], Wang et al. [35], and Pishchulin et al. [36]. The detailed results of the different datasets are tabulated in Table 1.

The overall performances of various approaches used in this paper are tabulated in Table 1. The performance results of our proposed model in terms of different poses and parameters are better than the existing methods with a small error of the model. The existing models shown in Table 1 only provide the human body joint points and the lines between the joint points as the body posture. The parameters used in existing schemes lack a lot of human body information and are not detailed and realistic enough. In contrast, the proposed model not only predicts the posture of the human body but also estimates the human body mesh model, so the proposed model is better than the existing schemes in overall prediction.

### 4.3. Experimental Results of Ablation Studies on Feature Extraction

The proposed model extracts two features of the Leeds Sports Pose (LSP) human posture image as the input of the model; in this section, we will analyze the impact of these features on the experiment. We have already discussed in detail the principles of HSV and TF functions, and here we have to analyze the influence of different combinations of these two characteristics.

We also conducted an experiment to verify the effectiveness of using dual input sources of TF and HSV features. In this experiment, when we use TF and HSV features as the input of CNN, we calculate the average accuracy (AP) of joint detection as shown in Table 2. On the LSP test dataset, using TF and HSV feature pairs can obtain better AP at all joints and the best mAP (average AP) at all joints. It is important to note that the TF and HSV features in this paper actually contain dual feature information. This is why, on the LSP, using only TF can lead to significantly better AP than using only HSV on the LSP test dataset. However, we standardize the body patch to a fixed size; the binary mask usually has a low resolution. As a result, we still need to combine TF and HSV features and construct a dual-channel CNN for pose estimation.

### 4.4. Experimental Results of Ablation Studies on Different Parameters

Considering that there are a large number of parameters that can be optimized in the network structure designed, the use of different parameter settings will have different effects on the accuracy and operating efficiency of the model. As a result, this paper conducts an ablation experiment analysis on different parameter configurations. Since the 3D pose estimation in this paper is implemented using a fully connected network with a varied number of neurons in the fully connected layer, the number of model parameters and the prediction effect are also different, so, in Figure 5, a different number of neurons (i.e., linear_size, representing the fully connected layer) is analyzed. The comparison of the loss function (loss curve of the number of neurons in) reveals that the loss value shows a gradual decay when the number of neurons increases from 256 to 4096. It indicates that the accuracy of the model training and the number of neurons are in a positive correlation. In other words, when the number of neurons increases, the model training is more convergent. Therefore, this paper further conducts a comparative experiment on the prediction effect of the network with different numbers of neurons. As shown in Figure 6, a batch of 50 test data pieces from the test set of Human 3.6 M is selected to verify the prediction effect of the model. The batch size is 64, and a total of 3200 test data pieces are used in this experiment. The abscissa in the figure represents the number of neurons in each layer, the parameters are set to 512, 1024, 2048, and 4096, and the ordinate represents the average value (mm) of node errors in the calculation of the batch of test data. By varying the number of neurons, the prediction result found that the error value of 4096 neurons is significantly lower than that of the 2048 neurons. Therefore, this paper sets the number of neurons in the fully connected layer to 4096. The convergence curves of different parameters are shown in Figure 7. The proposed model extracts two features of the LSP human posture image as the input of the model.

## 5. Conclusion

This paper proposes a novel action recognition model on the basis of deep neural network for football player action tracking and intervention. The proposed model extracts the texture and HSV features of the athlete's action image and proves the effectiveness of extracting these two features through ablation studies. The proposed model is to build a dual-channel convolutional neural network and prove its superiority through experimental results. The proposed model is capable of providing a scientific basis for the practitioners in the sports industry, especially the coaches, to formulate a reasonable training plan, thereby improving the level of football competition. Using the proposed model, not only athletes but also every individual will be physically active and strong.

## Figures and Tables

**Figure 1:** Example of footballer pose estimation and tracking.

**Figure 2:** The flowchart of the overall architecture of our AALI-Net algorithm.

**Figure 3:** Convolutional neural network.

**Figure 4:** Sliding window.

**Figure 5:** Convergence curves of different parameters.

**Figure 6:** The visualization results of football athlete training action recognition and tracking on the LSP dataset.

**Figure 7:** PCP comparison on LSP.

**Table 1:** PCP comparison on Leeds Sports Pose dataset using oks evaluation method.

Methods	Arm		Leg		Torso	Head
	Upper	Lower	Upper	Lower		
Dantone et al.	0.53	0.35	0.74	0.71	0.82	0.78
Tian et al.	0.45	0.38	0.52	0.69	0.81	0.65
Johnson et al.	0.52	0.31	0.64	0.52	0.71	0.74
Wang et al.	0.54	0.45	0.74	0.65	0.76	0.80
Pishchulin et al.	0.43	0.55	0.68	0.71	0.89	0.81
Proposed model	**0.81**	**0.61**	**0.85**	**0.82**	**0.90**	**0.85**

**Table 2:** Average precision of joint detection on LSP.

LSP	Ankle	Knee	Hip	Wrist	Elbow	Shoulder	Neck	Head	Map
*P*_TF_	0.25	0.34	0.23	0.23	0.43	0.32	0.21	0.34	0.31
*P*_HSV_	0.37	0.31	0.36	0.41	0.43	0.33	0.32	0.76	0.36
Proposed model	**0.45**	**0.42**	**0.45**	**0.31**	**0.43**	**0.54**	**0.58**	**0.79**	**0.47**

## Data Availability

The data used to support the findings of this study are included within the article.
